The article "Peroxisome Proliferator-Activated Receptor Gene Knockout Promotes Podocyte Injury in Diabetic Mice" was retracted in 2022. Reason: concerns about the peer review.

# Peroxisome Proliferator-Activated Receptor Gene Knockout Promotes Podocyte Injury in Diabetic Mice

**DOI:** 10.1155/2022/9018379

**Published:** 2022-06-30

**Authors:** Rui Yan, Ye Zhang, Yuxing Yang, Lingling Liu, Lirong Liu, Ziwei Guo, Haiyan Yu, Yuanyuan Wang, Bing Guo

**Affiliations:** ^1^Department of Nephrology Affiliated Hospital of Guizhou Medical University, Guiyang, 550004 Guizhou, China; ^2^Department of Endocrinology Affiliated Hospital of Guizhou Medical University, Guiyang, 550004 Guizhou, China; ^3^Guizhou Provincial Key Laboratory of Pathogenesis and Drug Research on Common Chronic Diseases, Guizhou Medical University, Guiyang, 550025 Guizhou, China; ^4^Department of Clinical Hematology, School of Clinical Laboratory Science, Guizhou Medical University, Guiyang, 550004 Guizhou, China

## Abstract

**Objective:**

To investigate the effects of peroxisome proliferator-activated receptor (PPAR*γ*) expression on renal podocyte in diabetic mice by conditionally knockout mouse PPAR*γ* gene.

**Methods:**

Wild-type C57BL mice and PPAR*γ* gene knockout mice were used as research objects to establish the diabetic mouse model, which was divided into normal control group (NC group), normal glucose PPAR*γ* gene knockout group (NK group), diabetic wild-type group (DM group), and diabetic PPAR*γ* gene knockout group (DK group), with 8 mice in each group. After 16 weeks, the mice were sacrificed for renal tissue collection. Morphological changes of renal tissue were observed by HE and Masson staining, and ultrastructure of renal tissue was observed by transmission electron microscope. Protein expressions of PPAR*γ*, podocin, nephrin, collagen IV, and fibronectin (FN) in renal tissues were detected by immunohistochemistry and Western blot, and mRNA changes of PPAR*γ*, podocin, and nephrin in renal tissues were detected by qRT-PCR.

**Results:**

Compared with the NC group, the protein and mRNA expressions of PPAR*γ*, podocin, and nephrin decreased in the kidney tissue of mice in the DM group, while the protein expressions of collagen IV and FN increased. The expression of various proteins in kidney tissues of the DK group was consistent with that of the DM group, and the difference was more obvious. The expression of PPAR*γ* protein and mRNA decreased in the NK group, while the expression of podocin, nephrin protein and mRNA, collagen IV, and FN protein showed no significant difference.

**Conclusion:**

In diabetic renal tissue, the loss of PPAR*γ* can aggravate podocellular damage and thus promote the occurrence of diabetic renal fibrosis. Increasing the expression of PPAR*γ* may effectively relieve renal podocyte impairment in diabetic patients, which can be used for the treatment of diabetic nephropathy.

The article "Peroxisome Proliferator-Activated Receptor Gene Knockout Promotes Podocyte Injury in Diabetic Mice" was retracted in 2022. Reason: concerns about the peer review.

## 1. Introduction

Diabetic nephropathy (DN) is a serious complication of diabetes [1, 2] and one of the main reasons that causes end-stage renal disease. Studies have shown that podocyte injury plays a very important role in the occurrence and development of diabetic nephropathy [3, 4].

Glomerulosclerosis is characterized by progressive proliferation of mesangial cells, deposition of extracellular matrix, and reduction of intrinsic glomerular cell composition. Podocytes, namely, the glomerular visceral epithelial cells, are attached to the lateral side of the glomerular basement membrane (GBM) and together with vascular endothelial cells and glomerular basal membrane constitute the glomerular filtration barrier [5, 6]. Podocytes have unique structures of foot processes, and abnormal expressions of the interconnecting slit diaphragm (SD) proteins nephrin, podocin, and CD2AP are characteristic markers of early injury of podocytes [7]. In 1998, Tryggvason discovered the podocyte slit diaphragm protein nephrin, which is specifically located in the podocyte slit diaphragm region and participates in maintaining the normal morphology and function of podocyte [8]. Podocin can form complex with nephrin to regulate the filtration permeability of filtered SD [9]. With the progression of DN, podocyte processes disappearance, fusion to sertoli cell apoptosis and abscission, destruction of glomerular basement membrane, and massive proteinuria may occur, and proteinuria itself may further aggravate podocyte injury, forming a vicious cycle, and eventually develop into end-stage renal disease [10–12].

Peroxisome proliferator-activated receptor *γ* (PPAR*γ*) is expressed in renal tubular epithelial cells, and its systemic activation has been shown to be protective against renal fibrosis [13]. The injury and shedding of podocyte are closely related to proteinuria, which is the key factor in the formation and development of glomerulosclerosis [14, 15]. Studies have found that pioglitazone, a peroxisome proliferator-activated receptor (PPAR*γ*) agonist, can reduce glomerular hypertrophy and glomerular hyperfiltration in KK/TA mice [16]. These results suggest that activation of PPAR*γ* is closely related to remission of DN [17, 18]. In addition, activation of PPAR*γ* has been documented to slow down podocyte damage and protect its integrity. Downregulation of PPAR*γ* expression in renal tubular epithelial cells also affects podocyte function [19]. However, the current study only observed the treatment of PPAR*γ* agonists and inhibitors, and the relationship between the expression changes of PPAR*γ* gene or protein itself in renal tissues and podocyte injury is not clear [20]. Therefore, this study intends to use conditional PPAR*γ* gene knockout diabetic mice as the research object and observe the expression changes of podocyte-related molecules in mouse kidney tissue after PPAR*γ* gene knockout.

The article "Peroxisome Proliferator-Activated Receptor Gene Knockout Promotes Podocyte Injury in Diabetic Mice" was retracted in 2022. Reason: concerns about the peer review.

## 2. Materials and Methods

### 2.1. Main Materials and Reagents

C57BL wild-type mice and C57BL renal tubule conditional PPAR*γ* gene knockout mice (SPF grade), with a body weight of 30 ± 5 g, were self-bred and identified (Professor Guan Youfei of Peking University Health Science Center presented a rat as a gift, SYXK (Beijing) 2011-0012). The following are the main materials and reagents: streptozotocin (STZ; SIGMA company); two-step immunohistochemistry detection reagent, horseradish peroxidase-labeled sheep anti-rabbit IgG, and DAB coloration kit (ZSGB Bio Co., Beijing); bicinchoninic acid protein concentration determination kit and ECL chromogenic agent (Beyotime Biotechnology, Beijing); prestained marker (Thermo Fisher Scientific); mouse anti-*β*-actin antibody (Bioworld, Nanjing); rabbit anti-PPAR*γ* antibody, rabbit anti-NPHS2 antibody, and rabbit anti-collagen-IV antibody (Proteintech); rabbit antinephrin antibody (Abcam); total RNA kit (TIANGEN Biochemical Technology Co., Beijing); real-time PCR assay kit (TaKaRa); and light microscopy and transmission electron microscopy (Precise, Beijing).

### 2.2. Establishment of Mouse DM Model and Experimental Grouping

Mice were randomly divided into 4 groups (the mice were presented by Professor Guan Youfei of Peking University Health Science Center): wild-type normal control group (NC), normal glucose PPAR*γ* gene knockout group (NK), wild-type diabetes group (DM), and diabetic PPAR*γ* gene knockout group (DK), with 8 mice in each group. For renal tubular epithelial cell conditional PPAR*γ* gene knockout mouse [21], triple loxE gene targeting strategy was adopted. Three loxP loci were introduced into the mouse PPAR*γ* gene to determine the DNA sequence of the PPAR*γ*^lox^ allele. Male mice heterozygous with the target allele (PPAR^w/lox + neo^) were crossbred with wild-type female mice to obtain single-celled embryos. Cre mediated partial or total recombination was achieved by microinjection of 0.1 ng/*μ*L Cre expressing plasmid (pBS185) into embryos. This resulted in the creation of wild-type (PPAR*γ*^W^) and knockout (PPAR*γ*^del^) PPAR*γ* allele mouse embryos, which were isolated by further reproduction.

The DM and DK groups received intraperitoneal injection of streptozotocin (STZ) (SIGMA company) 55 mg/(kg·day) for 5 days. After 2 weeks, tail venous blood was collected to measure blood glucose, and blood glucose above 16.7 mmol/L was considered as successful modeling. The mice in the four groups were fed to 16 weeks, fasted for 6 h, anaesthesia with ether, collected blood from femoral artery, and separated serum (centrifugation at 4°C). Blood glucose (BG) was measured by oxidase method. The kidneys were taken from both sides after laparotomy. One side was used for prepare paraffin sections (the kidney tissue was fixed in 4% paraformaldehyde) for pathological examination and immunohistochemical staining, and the other side was used for protein and RNA extraction (stored at -80°C) for Western blot and real-time PCR.

The article "Peroxisome Proliferator-Activated Receptor Gene Knockout Promotes Podocyte Injury in Diabetic Mice" was retracted in 2022. Reason: concerns about the peer review.

### 2.3. Immunohistochemical Test

PPAR*γ*, podocin, nephrin, collagen IV, and fibronectin proteins in renal tissues were determined by streptavidin-peroxidase (SP) two-step immunoassay kit. Paraffin sections of kidney tissues were dewaxed and hydrated and added 3% H_2_O_2_ to inhibit endogenous peroxidase. After microwave antigen repair, PPAR*γ* (1 : 200), podocin (1 : 250), nephrin (1 : 200), collagen IV (1 : 100), and fibronectin (1 : 50) specific primary antibodies were added and incubated overnight at 4°C. The next day, it was rewarmed to room temperature, rinsed, and incubated with secondary antibody (horseradish peroxidase labeled) for 30 min (37°C). Diaminobenzidine (DAB) was added for color rendering; hematoxylin was redyed, rinsed, dehydrated, and transparent; and the tablet was sealed with neutral gum. Leica microscope was used to randomly observe 5 fields at 200x magnification and collect images. The average number of stained cells was calculated for semiquantitative analysis.

Histopathological examination was performed by light microscopy and transmission electron microscopy at 400 times and 20000 times, respectively. Five visual fields were randomly selected for each group.

### 2.4. Western Blot

The cortical part of the kidney tissue was taken and added with histone lysate for full grinding; then, the supernatant was taken, and the protein concentration was determined with BCA protein detection kit (Beyotime Institute of Biotechnology, Beijing). Then, 50 ng supernatant was added into 2 × SDS sample buffer to prepare the sample. After fully mixing, the sample was bathed in water at 100°C for 10 min. Cool to room temperature, set aside at 4°C, or store at -20°C. After sample loading, electrophoresis, membrane transfer, and sealing, specific anti-PPAR*γ* (1 : 1000), anti-podocin (1 : 5000), anti-collagen-IV (1 : 500), anti-fibronectin (1 : 800) (Proteintech company), anti-nephrin (1 : 300) (Abcam), anti-*β*-actin (1 : 6000), (Bioworld Technology, Nanjing) were added, sealed, 4°C gently shake overnight. TBST was added to wash the membrane for 5 min × 3 times. The specific secondary antibody (ZSGB-Bio company) was incubated for 1 h, and the membrane was washed again with TBST for 5 min × 3 times. Add ECL (Beyotime Institute of Biotechnology, Beijing) development and exposure. Scans were performed using Shanghai Qinxiang gel imaging system. The ImageJ software analyzed the absorbance value of each band and detected the relative expression of each target protein, three times for each group.

The article "Peroxisome Proliferator-Activated Receptor Gene Knockout Promotes Podocyte Injury in Diabetic Mice" was retracted in 2022. Reason: concerns about the peer review.

### 2.5. Real-Time PCR

According to the kit instructions of TIANGEN Company, total RNA was extracted from renal tissues of mice in each group by TRIzol method. The cDNA was synthesized by reverse transcription-polymerase chain reaction with 20 *μ*L reaction system. Primers for PPAR*γ*, podocin, and nephrin mRNA were synthesized by Shanghai Sangon Biotech Co., Ltd. Primer sequences are shown in Table 1. TB Grenn™ Premix Ex Taq™ II (Takara) was used for quantitative PCR. The experiment was repeated three times for each group.

### 2.6. Statistical Treatment

The experimental data were processed and analyzed by the GraphPad Prism 5 and SPSS 19.0 softwares. Mean ± SD ($\bar{x}\pm s$) was used to represent measurement data. After the data passed the test of variance, one-way ANOVA was used between multiple groups, and least significant difference (LSD) method was used to analyze and compare the two groups of samples. When *P* < 0.05, the difference was statistically significant.

## 3. Results

### 3.1. General Situation and Biochemical Indexes of Mice

After the replication of the DM model induced by STZ, mice in the DM and DK groups showed polydipsia, polyphagia, polyuria, and weight loss. Compared with the NC group or NK group, blood glucose (*P* < 0.01), blood creatinine, and blood urea nitrogen (*P* < 0.05) in the DM and DK groups were increased. Compared with the DM group, the increase of above indexes in the DK group was more significant, but the difference was not statistically significant, as shown in Table 2.

### 3.2. Renal Histomorphology

The renal tissues of mice were examined by pathological examination. HE staining showed complete glomerular morphology, no dilation and necrosis of renal tubules, and complete basement membrane of mice in the NC and NK groups. In the DM group, the lumen of renal tubules was dilated, the epithelial cells were swollen and vacuolated, the basement membrane was irregular thickened, and there were many inflammatory cells infiltrating in the interstitium. The above changes were more obvious in the DK group. Masson staining showed no collagen deposition in the glomerular basement membrane, mesangial area, and interstitial area of renal tubules in the NC and NK groups. The above changes were more serious in the DK group, presenting extensive fibrosis (Figure 1(a)). Transmission electron microscopy showed that the renal ultrastructure was normal in the NC group and NK group. The basement membrane of glomerular capillaries was thickened and mesangial matrix was increased structural changes of podocytes, extensive fusion of foot processes, and increase of hiatus between foot processes were observed in renal tissues of the DM and DK groups (Figure 1(b)).

The article "Peroxisome Proliferator-Activated Receptor Gene Knockout Promotes Podocyte Injury in Diabetic Mice" was retracted in 2022. Reason: concerns about the peer review.

### 3.3. Expression of PPAR*γ* Protein in Renal Tissues of Each Group

The expression levels of PPAR*γ* protein in kidney tissues of mice in four groups were detected by immunohistochemistry and Western blot. Immunohistochemical results showed that PPAR*γ* was highly expressed in renal tissues of mice in the NC group, and the staining result was strongly positive (+++). The expression level of PPAR*γ* protein in the NK group and DM group was lower than that in the normal group, and the staining result was medium positive (++). The protein expression level was lowest in the DK group, and the staining result was weakly positive (+) (Figure 2(a)). WB results were consistent with immunohistochemical results (Figure 2(b)). qRT-PCR results showed that compared with the NC group, PPAR*γ* mRNA levels in the NK, DM, and DK groups were decreased, and the differences were statistically significant (∗*P* < 0.05). Compared with the DM group, PPAR*γ* mRNA level in the DK group was significantly lower (#*P* < 0.05) (Figure 2(c)).

### 3.4. Podocin and Nephrin Protein Expressions in Renal Tissues of Each Group

Immunohistochemical results showed that podocin staining was strongly positive (+++) and nephrin staining was moderately positive (++) in the NC group. NK group podocin and nephrin staining results were medium positive (++). Podocin and nephrin staining results were weakly positive (+) in the DM group. Podocin and nephrin staining results were negative in the DK group (Figure 3(a)). qRT-PCR results showed that compared with the NC group, the mRNA levels of podocin and nephrin in the DM group were decreased, and the expression level of podocin and nephrin in the DK group was the lowest; the difference was statistically significant (∗*P* < 0.05, ∗∗*P* < 0.01). No significant difference was found in the NK group (*P* > 0.05) (Figure 3(b)). The results of Western blotting showed that podocin and nephrin were highly expressed in renal tissues of the NC group and NK group, while the expression levels of podocin and nephrin in the DM and DK groups were lower than those in the NC group. Compared with the DM group, the protein expression level of the DK group was the lowest (Figure 3(c)).

The article "Peroxisome Proliferator-Activated Receptor Gene Knockout Promotes Podocyte Injury in Diabetic Mice" was retracted in 2022. Reason: concerns about the peer review.

### 3.5. Protein Expression of Collagen IV and Fibronectin in Renal Tissues of Each Group

Immunohistochemical results showed that the staining results of the NC group and NK group were the same: collagen IV and fibronectin staining were negative. Collagen IV and fibronectin staining were weakly positive (+) in the DM group. In the DK group, collagen IV staining was strongly positive (+++), and fibronectin staining was moderately positive (++) (Figure 4(a)). WB results showed that the expression levels of collagen IV and fibronectin in renal tissues of the NC group and NK group were very low, and the expression levels of collagen IV and fibronectin in the DM group and DK group were higher than those in the normal group (∗*P* < 0.05, ∗∗*P* < 0.01), and the protein expression level of the DK group was the highest (Figure 4(b)).

## 4. Discussion

The pathological changes of diabetic nephropathy mainly include glomerulosclerosis and tubulointerstitial fibrosis [22]. The main pathological processes of renal interstitial fibrosis include changes in tissue microenvironment caused by renal injury, myofibroblast activation and proliferation, production and deposition of a large amount of extracellular matrix (ECM), renal tubular atrophy, and capillary loss [23]. ECM is a noncellular scaffold structure located in the renal interstitium, which provides physical support for renal tubules and capillaries and regulates tissue homeostasis under physiological conditions [24]. ECM is rich in fibrin, matrix proteins, proteoglycans, and other cytokines that promote fibrosis [25]. Fibrin forms the framework of ECM and is the main component of ECM. Fibrin mainly includes collagen, fibronectin, and elastin. Therefore, these protein changes can be a marker of fibrotic lesions.

A large number of studies have confirmed that PPAR*γ* receptor agonists have a significant renal protective effect in the treatment of DN. Choi et al. [26] found that the phosphorylation of PPAR*γ* mediated by cyclin-dependent kinase 5 (Cdk5) may be involved in the pathogenesis of insulin resistance, while rosiglitazone can block the phosphorylation of CK5-PPAR. This inhibition is effective both in vivo and in vitro. Meanwhile, rosiglitazone has significant antidiabetic effects [27] and insulin sensitization [28]. It has been proved that the expression of PPAR*γ* in NRK-52E cells was inhibited and phosphorylated in high glucose environment, but no such changes occurred in mannitol environment [29]. And PPAR*γ* agonist can effectively protect podocyte and regulate podocyte injury [30].

Therefore, in order to investigate the correlation between the expression of PPAR*γ* in mouse renal tissue and podiocytes injury, this study used renal tubular epithelial cell conditioned PPAR*γ* gene knockout mice, and intraperitoneal injection of STZ was used to replicate the normal wild mice and the DN model of PPAR*γ* knockout mice. Subsequently, the changes of renal tissue structure were observed by light microscope and electron microscope, and the protein and mRNA expressions of PPAR*γ*, podocin, nephrin, collagen IV, and fibronectin were detected by immunohistochemistry, Western blot, and real-time PCR. Under light microscope, the renal tubule lumen of mice in the DM group and DK group was dilated, epithelial cells were swollen and vacuolated, basement membrane was irregular thickened, and there were many inflammatory cells infiltrating in the interstitium. The above changes were more obvious in the DK group. The glomerular mesangial matrix was increased, and the foot process was fused extensively under electron microscope. In protein level detection, it was found that the expression levels of PPAR*γ*, podocin, and nephrin in renal tissue of mice in the DN group were decreased, accompanied by upregulated expressions of collagen IV and fibronectin; markers of renal interstitium fibrosis and the above protein expression changes were more obvious in renal tissue of mice in the DK group. However, there was no statistical significance in the NK group. In conclusion, PPAR*γ* deletion promoted podocyte injury and aggravated DN fibrosis in DN condition, while in normal glucose condition, PPAR*γ* deletion did not cause obvious podocyte injury and renal fibrosis, which may be related to the absence of PPAR*γ* phosphorylation. Meanwhile, mRNA changes of PPAR*γ*, podocin, and nephrin were consistent with protein level changes. In conclusion, in DN mouse kidney tissue, PPAR*γ* deletion can reduce the expression of podocyte marker protein podocin and nephrin and aggravate the occurrence of renal fibrosis.

The article "Peroxisome Proliferator-Activated Receptor Gene Knockout Promotes Podocyte Injury in Diabetic Mice" was retracted in 2022. Reason: concerns about the peer review.

In this study, we elucidated the changes of PPAR*γ* and Podocyte marker expression in mouse renal tissue under DN condition and their relationship with renal fibrosis. However, there are still some deficiencies in this study. It is not clear how PPAR*γ* regulates podocyte injury. In the future, we will further study specific regulatory links and mechanisms from in vitro and clinical trials.

## Figures and Tables

**Figure 1:** (a) Pathological examination of renal tissues of mice in each group by light microscopy (400x). (b) The ultrastructure of renal tissue was observed by transmission electron microscope (20,000x).

**Figure 2:** (a) The expression of PPAR*γ* in renal tissues of each group was detected by immunohistochemistry (400x). (b) The expression of PPAR*γ* was detected by WB. (c) The expression of PPAR*γ* was detected by RT-qPCR. Compared with the NC group, ^∗^*P* < 0.05 and ^∗∗^*P* < 0.01. Compared with the DM group, #*P* < 0.05.

**Figure 3:** (a) The expression of podocin and nephrin in renal tissues of each group was detected by immunohistochemistry (SP assay, 200x). (b) WB detected the expression of podocin and nephrin in tissues. (c) RT-qPCR detected the expression of podocin and nephrin in tissues. Compared with the NC group, ^∗^*P* < 0.05 and ^∗∗^*P* < 0.01. Compared with the DM group, #*P* < 0.05.

**Figure 4:** (a) The expression of collagen IV and fibronectin in renal tissues of each group was detected by immunohistochemistry (SP assay, 200x). (b) WB detected the expression of collagen IV and fibronectin in tissues. Compared with the NC group, ^∗^*P* < 0.05 and ^∗∗^*P* < 0.01. Compared with the DM group, #*P* < 0.05.

**Table 1:** Primer sets used in real time RT-PCR.

Gene	Upstream primer	Reverse primer
PPAR*γ* Podocin Nephrin	5′-TTTCAAGGGTGCCAGTTTCG-3′ 5′-TGAGGATGGCGGCTGAGAT-3′ 5′-CCCAACACTGGAAGAGGT-3′	5′-ATCCTTGGCCCTCTGAGATGAG-3′ 5′-GGTTTGGAGGAACTTGGGT-3′ 5′-CTGGTCGTAGATTCCCCTTG-3′
*β*-Actin	5′-GCTACAGCTTCACCACCACA-3′	5′-AAGGAGGCTGGAAAAGAGC-3′

**Table 2:** Biochemical indexes of mice.

Index	NC	NK	DM	DK
Weight (g)	31.0 ± 2.3	30.3 ± 2.5	29.6 ± 4.3	25.6 ± 5.2^∗^
Blood glucose (mmol/L)	12.3 ± 1.4	11.0 ± 2.9	33.6 ± 12.1^∗∗^	32.2 ± 6.9^∗∗^
Blood creatinine (*μ*mol/L)	10.2 ± 2.5	13.5 ± 3.2	17.3 ± 2.5^∗^	18.7 ± 4.0^∗^
Blood urea nitrogen (mmol/L)	6.9 ± 1.2	8.1 ± 1.7	13.9 ± 3.4^∗^	16.7 ± 3.2^∗^

Note: ^∗^*P* < 0.05; ^∗∗^*P* < 0.01.

## Data Availability

The datasets used and/or analyzed during the current study are available from the corresponding authors on reasonable request.
